The article "Design of Fuzzy Aided Cognition System for International Economic and Trade Information under Supply Chain Management" was retracted in 2022. Reason: concerns about the peer review.

# Design of Fuzzy Aided Cognition System for International Economic and Trade Information under Supply Chain Management

**DOI:** 10.1155/2022/6516175

**Published:** 2022-02-02

**Authors:** Donghong Ren, Zamira Madina

**Affiliations:** ^1^School of Economics and Management, Shangqiu Polytechnic, Shangqiu 476000, China; ^2^The Department of Industrial Engineering, International Ataturk Alatoo University, Kyrgyzstan

## Abstract

The existing fuzzy assistant cognition system has the problem of imperfect retrieval function, which leads to long execution time. This paper designs a fuzzy assistant cognition system of international economic and trade information under supply chain management. *Hardware Part*. Optimize wireless sensor and connect power interface and related accessories. In the software part, the dynamic characteristics of international economic and trade information elements are extracted, the flexible operation model of supply chain management is constructed, the demand-oriented organizational structure is established, the output set is determined by the product reasoning, and the retrieval function of fuzzy assistant cognitive system is designed by using the fuzzy association algorithm. *Experimental Results*. The average execution time of the fuzzy assistant cognitive system and the other two systems is 123.593 s, 165.733 s, and 169.506 s, which proves that the cognitive system integrated with supply chain management has a higher practical application value.

## 1. Introductions

Supply chain is divided into internal supply chain and external supply chain. Earlier, it was the view of internal supply chain: supply chain is an internal process in manufacturing enterprises, which refers to the supply and demand process composed of purchasing department, production department, and storage department involved in the internal product production and circulation process [1–3]. This notion is restricted to the enterprise's internal operations, focused on the utilization of its own resources. The notion of an external supply chain considers the supply chain's external environment. It is the conversion of raw materials into products via the processing of various firms in the supply chain and subsequently to end customers. It is a more expansive and global notion. All operations connected to the manufacturing and distribution of goods from suppliers to consumers are included in supply chain management. The four core processes of supply chain management are described first in this definition: planning, buying, production, and distribution. At the same time, it stresses the breadth of supply chain management, implying that it is a management activity that spans companies and numerous functional groups [4, 5]. An empirical study on the link between international commerce and economic development has grown in importance during the last half-century. Prior to the 1960s, most studies on trade and economic development were restricted to basic comparative studies of a few representative nations. However, since various economists use different models and research methodologies, their results are often varied. However, due to different models and research methods adopted by different economists, their conclusions are quite different. The domestic and foreign research results on international economy and trade mainly focus on the following five aspects: trade promoting economic growth, export promoting economic growth, import promoting economic growth, trade policy and economic growth, and the mechanism of trade promoting economic growth, and on this basis, the use of modern measurement methods for research [6–8]. With the advancement of science and technology, as well as the arrival of the big data era, it is becoming increasingly important to realize cognition and judgment similar to that of the human brain, to discover new relevance and fuzzy auxiliary cognitive modes, and to make correct decisions, all of which present new opportunities and challenges for cognitive computing technology development. To overcome this challenge, it is critical to understand how to employ cognitive computing, a relatively recent computing mode technology, to break past old technological barriers and construct a fuzzy auxiliary cognitive system. At present, the academic literature on the fuzzy assistant cognitive system of supply chain management and international economic and trade information is not very rich, which needs to be further explored.

The article "Design of Fuzzy Aided Cognition System for International Economic and Trade Information under Supply Chain Management" was retracted in 2022. Reason: concerns about the peer review.

## 2. Hardware Design of Fuzzy Aided Cognition System for International Economic and Trade Information under Supply Chain Management

Wireless sensor network configuration, in wireless sensor network, nodes in the network can be divided into full function devices and reduced function devices according to the communication ability of node devices. Following the successful establishment of the wireless sensor network, all nodes interact according to the following rules: FFD and RFD can connect with each other; however, RFD can only communicate with FFD, which means that the coordinator sends orders to the control node or the control node returns the gathered data information to the coordinator. The quantity of data conveyed by RFD is smaller due to the necessity of low power consumption and therefore uses less transmission and communication resources. It is mostly utilized for data gathering and basic control applications. The network may be classified as a star network, mesh network, or cluster network depending on the networking environment. All devices communicate with the central device in the star structure, and the communication unit is routed. Any two FFD devices in a mesh network can communicate directly with a specific protocol as long as they are within the effective range of each other's wireless radiation, and each FFD device in the mesh network can become a network router to realize the function of network packet routing and forwarding. It is more difficult to construct a mesh network than a star network because mesh nodes must keep more information. A cluster network is a more complicated topology made up of numerous basic star networks that may be expanded by a complex star network. However, as compared to the creation of a mesh network, the creation of a cluster network needs fewer resources. A node is a device that corresponds to a wireless MCU such as the CC2530: each device has a wireless radio terminal and an IEEE address and network address that is unique. To construct a genuinely dispersed control network, typical wireless sensor nodes may provide interdisciplinary characteristics and functions. The power module, processor module, sensor module, and wireless communication module are the four primary components of a wireless sensor network node [9]. The CC2530 chip has an 8051 single-chip processor that combines the wireless communication module with the CPU module. Then, as illustrated in Figure 1, the whole node hardware design may be condensed into three primary elements.

The design scheme creates a wireless sensor network using a series of sensor modules and wireless node modules, extends the embedded gateway to achieve wide-area access, realizes wireless sensor network networking, and configures sensor data collection, wireless signal receiving and sending, network communication, and the entire component control and network communication process. By employing cluster ID, the device binding procedure establishes a logical connection for various unique endpoints. The following steps are involved in binding: first, the endpoint must send binding requests to the coordinator; second, the coordinator must receive binding requests from two endpoints within a specific time interval in order to establish a binding table between the endpoints; and finally, the coordinator must form a specific logical link between the endpoints in the binding table. Following that, you may send direct and indirect messages between the two bound endpoints. The binding endpoints communicate in the following way: initially, one of the endpoints sends information to the coordinator node. The coordinator node looks up the binding table after receiving the message and then sends the message to all the endpoints bound to this endpoint to complete the communication. When the RFD device wishes to transmit data frames to the FFD device in a star network without a beacon, it just has to wait for the channel to become idle before sending the data frames. The hardware design of the fuzzy assistant cognition system has been finished based on the preceding description.

The article "Design of Fuzzy Aided Cognition System for International Economic and Trade Information under Supply Chain Management" was retracted in 2022. Reason: concerns about the peer review.

## 3. Software Design of Fuzzy Assistant Cognition System for International Economic and Trade Information under Supply Chain Management

### 3.1. Extracting the Dynamic Characteristics of International Economic and Trade Information Elements

It can be seen that the research on international economic and trade information can be carried out through two dimensions, one is the long-term impact, the other is the short-term impact. In the short run, three factors jointly determine a country's economic growth, namely, investment demand, consumption demand, import, and export. The scenario will grow considerably more difficult in the long term. Increases in capital and labor, on the other hand, lead to the buildup of economic strength. This study examines the three processes of capital accumulation, technical innovation, and institutional innovation, starting with the long-term impact. From the standpoint of material capital, we discovered that there was a strong association between capital accumulation and economic expansion in the early twentieth century, implying that capital accumulation was the major element in promoting economic progress [10, 11]. Capital accumulation, according to the Solow model, will raise per capita capital stock, causing a country's output to grow. Assuming that the saving rate stays constant, per capita production will rise, boosting a country's economic development. International trade mostly promotes economic development by increasing capital accumulation in the following three conditions. Because there are too many researches on the index of natural resources, we choose capital (including labor and material capital), technology, and institutional factors to study. The expression formula of natural resource factors is as follows:

(1) $$\begin{array}{c} R=y-\left(y+e\right)\alpha . \end{array}$$

In formula (1), *y* is the total economic volume in a year, *e* is the rate of trade, and *α* is the stock proportion of trade products. Due to the role of international trade, the export of foreign products will make domestic export enterprises face more competitive environment. Enterprises must improve capital accumulation, hold more acquired cash for a longer length of time, become the driving force of investment demand, and boost development if they are to survive. Furthermore, economies of scale and competitive advantage are essential considerations. According to the theory of factor endowments, if the government does not intervene directly, the enterprise can import and export directly, indicating that the product produced by the enterprise has a comparative advantage, and it can also be put into production and export trade for this kind of product, resulting in comparative advantage benefits [12–14]. At the same time, there is a benefit in that after exporting items with comparative advantages, certain businesses may split and occupy international market share. When the two areas' trade situation approaches equilibrium, real consumption equals actual production. The utility flow is the logarithmic form of the actual consumption. Therefore, the indirect utility function is the economic growth rate; the specific expression formula is as follows:

(2) $$\begin{array}{c} \log\left(k\right)=\frac{D}{\delta }\times k. \end{array}$$

In formula (2), *D* is the utility flow, *δ* is the given economic change, and *k* is the economic growth rate. The results of formula (2) can show that the accumulation of enterprise capital can improve the profit rate of enterprises, and thus, the capital accumulation rate can be improved, which will ultimately promote economic growth. In development economics, there is a classic theory and model, namely, “vicious circle of poverty” theory and Harold Domar model. The study believes that the level of saving rate is a major reason for economic growth [15]. However, according to the above assumption, the national saving rate in emerging nations after WWII is quite high, but it does not contribute to capital accumulation. Many variables may contribute to the aforementioned issue, but the fundamental explanation must be a lack of investment opportunities in these nations. A nation may enhance economic development by continuously accumulating capital if it can attract more foreign investment and improve the investment climate. The dynamic properties of international economic and trade data items are retrieved based on this.

The article "Design of Fuzzy Aided Cognition System for International Economic and Trade Information under Supply Chain Management" was retracted in 2022. Reason: concerns about the peer review.

### 3.2. Construction of Flexible Operation Model for Supply Chain Management

The operating method of supply chain management may free the interchange of products and information from the constraints of time and place. Anyone can use the e-commerce service function to conduct relevant e-commerce activities at any time and from any location, and businesses can use the network to expand their scope of business activities to the entire world; consumers can choose the goods and services they want from anywhere on the planet. Customers' preferences for product kinds and service quality are becoming more individualized. Supply chain management theory and methods are developed in the context of current science and technology. The basic techniques of supply chain management in the information age include quick response, effective user response, e-commerce, and just-in-time manufacturing [16, 17]. In the process of trade, the calculation formula of enterprise return under supply chain management is as follows:

(3) $$\begin{array}{c} w=h\times \overset{u}{\underset{m}{\sum }}S. \end{array}$$

In formula (3), *h* is the accumulated trade volume, *S* is the trade input, *u* is the enterprise return value, and *m* is the labor demand. There is a high degree of uncertainty in the supply chain management, from the market situation, the changing consumer demand to the internal operation management of the system, which are the management difficulties. Some of the factors can be resolved through human efforts, while others are unpredictable, so we can only take some measures and design the corresponding management mode to avoid them, to achieve the best results. Then, the expression formula of enterprise economic growth value is as follows:

(4) $$\begin{array}{c} Q=\frac{1}{v}\varphi^{-1/2}. \end{array}$$

In formula (4), *v* is the trade risk and *φ* is the rising space of capital. Based on the theory of flexibility, flexible management realizes flexible and agile operation mechanism by improving the flexibility of various resources and improves the market competitiveness of enterprises with flexible organization management, flexible personnel, and flexible production system. In the environment of supply chain management, the application of flexible strategy will make the operation of the system more able to adapt to the rapidly changing market demand [18, 19]. On the basis of formula (4), the conditions for enterprises to reach equilibrium in the capital market under supply chain management are obtained; the specific expression formula is as follows:

(5) $$\begin{array}{c} \frac{d}{F_{\varepsilon }}+\frac{\varepsilon }{P_{\varepsilon }}=F+P. \end{array}$$

In formula (5), *F* is the normal interest rate of the enterprise, *P* is the proportion of investment in total assets, *d* is the jump variable, and *ε* is the proportion of investment. To create a flexible supply chain, we must first start at each node, develop a demand-driven enterprise strategy and organizational structure, implement advanced production and management technology, improve information sharing and communication among various departments within the enterprise, and continuously improve the strength and flexibility of each enterprise. Second, to prevent difficulties in the supply chain's connecting link, it is vital to enhance the connection between each node, develop a reliable information exchange platform, and pick suppliers with a strong reputation and competitive advantage for collaboration. Finally, all supply chain enterprises should have a global perspective, analyze and solve supply chain problems from a system theory perspective, and collaborate to promote effective information sharing and accelerate logistics distribution speed, in order to make the supply chain operate efficiently. Based on the above description, the steps of building a flexible operation model are completed.

The article "Design of Fuzzy Aided Cognition System for International Economic and Trade Information under Supply Chain Management" was retracted in 2022. Reason: concerns about the peer review.

### 3.3. Design of Retrieval Function of Fuzzy Assistant Cognitive System Based on Fuzzy Association Algorithm

There are various fuzzy assistant cognitive system learning methods, but they are all based on a semifuzzy model, in which the fuzzy membership function of the premise is a single value [20]. In the presence of noise, the single-valued fuzzy generating approach is ineffective. A comprehensive fuzzy model learning technique based on the steepest descent approach is presented in this study. The fuzzy association method analyzes the various target feature information from the main sensor and each auxiliary sensor to deliver the association pairing table between the point trace and the track if the output fuzzy set is defined by product reasoning. It is clear that the system makes use of a range of feature data to increase data association quality while keeping the tracking filter as simple as feasible. Only relevant feature information, such as distance, velocity, acceleration, target movement direction, and radial velocity, is considered for the purpose of simplicity. The introduction of radial velocity data has been thoroughly examined [21–23]. But the extraction of radial velocity requires a nonlinear motion model and nonlinear filtering method, which increases the complexity of the system. The radial velocity feature can be extracted from pulse-Doppler radar data; the expression formula of Doppler translation is as follows:

(6) $$\begin{array}{c} q\left(\phi \right)=\left(\frac{2}{\phi }\right)L\left(\phi \right). \end{array}$$

In formula (6), *ϕ* is the speed of information propagation and *L* is the wavelength of the transmitted wave. The information retrieval module is responsible for retrieving the relevant information from the question answering knowledge base and transferring it to the subsequent answer generation and processing module. Based on different types of user problems, the retrieval data form of the system is also different. The importance of target motion direction information is that its first derivative is angular velocity to represent the change of target motion direction. It is very important to judge the association when multiple targets cross. The direction feature information can be obtained from the position measurement data, but due to the existence of noise, it is necessary to find a feasible statistical estimation method. Based on the maximum likelihood direction estimation method, the expression formula of target information trajectory measurement value is obtained as follows:

(7) $$\begin{array}{c} V=\frac{\sqrt{\left(f^{2}+4\eta \right)}}{2}. \end{array}$$

In formula (7), *f* is the Gaussian random variable, and *η* is the measured value of the data point. For the questions based on question-answer pairs, the fuzzy assistant cognitive system can get answers by connecting the results of deep language analysis with a knowledge map. For the problem based on free-text data, information retrieval is directly through Turing knowledge base query [24]. Based on the retrieval information obtained from information retrieval, the answer generation module of the cognitive system mainly realizes the extraction of candidate answers and the calculation of confidence degree of answers and finally returns concise and correct answers. According to the granularity of answer information, candidate answer extraction can be divided into paragraph answer extraction, sentence answer extraction, and phrase answer extraction. The calculation formula of fine-grained information is as follows:

(8) $$\begin{array}{c} \beta =\frac{1}{G-1}\underset{i=1}{\sum }N. \end{array}$$

In formula (8), *G* is the track value of data point, *N* is the input characteristic information, and *i* is the information deviation. According to the data domain of the user's question, the question types can be divided into domain-oriented questions, open domain-oriented questions, and common problem sets. According to the different data sources of answers, answers can be divided into structured-data-based answers, free-text-based answers, and question and answer pair-based answers. Different types of questions and answers have different methods for data processing. Based on this, the retrieval function of the fuzzy assistant cognitive system is designed.

The article "Design of Fuzzy Aided Cognition System for International Economic and Trade Information under Supply Chain Management" was retracted in 2022. Reason: concerns about the peer review.

## 4. Experimental Test

### 4.1. Setting Up Experimental Environment

Experiment with the design system and develop the experimental environment to ensure its efficacy. The platform's deployment mechanism is built based on the platform's and database's properties. The distributed deployment option is used by the intelligent cognitive system, which uses 11 servers. The particular cognitive computing database supports intention and question answering queries, whereas sol offers a search engine, HBase gives rapid random access to vast structured data, and Neo4j provides data support. A public opinion web crawler provides the current news information, and the platform uses a unified basic map service. The intelligent cognitive system and database are supported by the hardware-operating environment, which includes a database server, application server, business management application front-end computer, data backup equipment, and printing equipment. The auxiliary cognitive system's web server uses the virtualization server, while the application server uses the Internet of Things cloud platform's current application server architecture. Other hardware facilities combine and use the Internet of Things cloud platform project's current hardware resources rather than purchasing new hardware. The software environment consists mostly of the R&D environment for software, the server operating system, and numerous business support tools. Environment for R&D: based on JDKL. 7 and above, Tomcat 7 and above, including database management software, J2EE application server, GIS software, Turing machine man, synonym API, cloud API, MySQL database, etc. In the above experimental environment, the experimental test is carried out and the experimental results are obtained.

### 4.2. Experimental Result

In the experiment, the MVC-based fuzzy assistant cognitive system and the metacognition-based fuzzy assistant cognitive system are selected to test with the designed fuzzy assistant cognitive system. Under different number of data exchange request tasks, the less the execution time of the three systems, the better the system performance. The experimental results are shown in Tables 1–3.

According to Table 1, the average execution time of the fuzzy assistant cognitive system is 83.305 s, 115.265 s, and 113.298 s compared with the other two systems. According to Table 2, the average execution time of the fuzzy assistant cognitive system is 127.831 s, 161.01 s, and 164.271 s. According to Table 3, the average execution time of the designed fuzzy auxiliary cognitive system and the other two systems is 159.645 s, 220.926 s, and 230.95 s, which indicates that under the same experimental conditions, the designed system is more suitable for the auxiliary cognitive scene.

## 5. Conclusions

The design of the auxiliary cognitive system enriches the academic literature on supply chain management and fuzzy auxiliary cognitive system and provides new feasible ideas for related research. At the same time, it broadens the application scope of fuzzy assistant cognitive system and lays a theoretical and practical foundation for the follow-up research. Due to the limited research conditions, the accuracy of the design system has not been verified in this paper. In the future, we will continue to work on related research and make continuous progress.

The article "Design of Fuzzy Aided Cognition System for International Economic and Trade Information under Supply Chain Management" was retracted in 2022. Reason: concerns about the peer review.

## Figures and Tables

**Figure 1:** Hardware node module.

**Table 1:** Execution time of 50 data exchange request systems (s).

Number of experiments	Fuzzy assistant cognition system based on MVC architecture	Fuzzy assistant cognition system based on metacognition	Fuzzy aided cognitive system for design
1	112.41	99.87	85.66
2	109.38	105.22	88.14
3	123.47	116.34	79.68
4	106.19	126.44	81.02
5	123.56	105.74	82.74
6	116.58	126.18	82.59

**Table 2:** Execution time of 100 data exchange request systems (s).

Number of experiments	Fuzzy assistant cognition system based on MVC architecture	Fuzzy assistant cognition system based on metacognition	Fuzzy aided cognitive system for design
1	156.32	161.05	131.08
2	162.47	168.55	126.09
3	169.33	171.69	125.77
4	159.64	165.22	132.69
5	153.02	158.87	128.54
6	165.28	160.25	122.82

**Table 3:** Execution time of 200 data exchange request systems (s).

Number of experiments	Fuzzy assistant cognition system based on MVC architecture	Fuzzy assistant cognition system based on metacognition	Fuzzy aided cognitive system for design
1	225.41	246.55	165.37
2	216.39	239.16	162.47
3	207.44	220.11	159.36
4	226.19	239.91	148.22
5	237.66	206.38	163.17
6	212.47	233.59	159.28

## Data Availability

Data are available on request.
